The article "Rho GTPase-activating protein 35 suppresses gastric cancer metastasis by regulating cytoskeleton reorganization and epithelial-to-mesenchymal transition" was published in 2022. Journal: Bioengineered.

# Rho GTPase-activating protein 35 suppresses gastric cancer metastasis by regulating cytoskeleton reorganization and epithelial-to-mesenchymal transition

**DOI:** 10.1080/21655979.2022.2092677

**Published:** 2022-06-26

**Authors:** Yi Sun, Rui Du, Yulong Shang, Changhao Liu, Linhua Zheng, Ruiqing Sun, Yuanyong Wang, Guofang Lu

**Affiliations:** a Department of Ultrasound Diagnostics, Tangdu Hospital, Fourth Military Medical University, Xi’an, shaanxi, China; b Institute for Biomedical Sciences of Pain, Tangdu Hospital, Fourth Military Medical University, Xi’an, shaanxi, China; c State Key Laboratory of Cancer Biology and National Clinical Research Center for Digestive Diseases, Xijing Hospital of Digestive Diseases, Fourth Military Medical University, Xi’an, shaanxi, China; d Department of Radiation Oncology, Xijing Hospital, Fourth Military Medical University, Xi’an, shaanxi, China; e Department of Thoracic Surgery, Tangdu Hospital, Fourth Military Medical University, Xi’an, shaanxi, China; f Department of Physiology and Pathophysiology, National Key Discipline of Cell Biology, Fourth Military Medical University, Xi’an, Shaanxi, China

**Keywords:** ARHGAP35, metastasis, cytoskeleton, gastric cancer, Epithelial-mesenchymal transition

## Abstract

Cytoskeletal reorganization and epithelial-to-mesenchymal transition (EMT) are key processes and typical characteristics of metastatic cancer cells. Rho GTPase‑activating protein 35 (ARHGAP35) is a GTPase-activating protein, which has a significant effect on cell motility. However, the particular function of ARHGAP35 in gastric cancer (GC) remains unknown. In the present study, the role of ARHGAP35 in GC was investigated by *in vitro* loss-of-function and gain-of-function experiments. Cytoskeletal reorganization in GC cells was evaluated using immunofluorescence staining and the protein expression levels of key molecules and active RhoA were detected by western blot analysis. Additionally, the clinical evaluation of proteins in human GC tissues was assessed by immunohistochemistry. The results showed that ARHGAP35, a tumor suppressor, was downregulated in GC tissues and its decreased expression was associated with the metastatic status of GC. Additionally, Transwell and wound healing assays demonstrated that ARHGAP35 knockdown promoted cell motility *in vitro*. However, the above effects were abrogated following ectopic ARHGAP35 expression. Furthermore, ARHGAP35 could affect cytoskeletal reorganization via directly regulating RhoA activation. In addition, ARHGAP35 upregulated E-cadherin and attenuated EMT in GC cells. Both ARHGAP35 and E-cadherin were associated with overall survival in patients with GC, while their combination allowed for an even greater capacity for distinguishing GC patients with different prognosis. Overall, the results of the current study suggested that ARHGAP35 could directly regulate cell morphology and motility via affecting cytoskeletal reorganization and EMT via targeting RhoA and E-cadherin, respectively. Targeting the ARHGAP35/RhoA/E-cadherin pathway could be a potential approach for treating GC.

## Highlights

- Epithelial-to-mesenchyma transition was re-stored following ARHGAP35 overexpression.
- ARHGAP35 could directly regulate cell cytoskeleton reorganization via activating RhoA.
- ARHGAP35/RhoA/E-cadherin axis could be a potential treatment approach for GC.

## 1. Introduction

Gastric cancer (GC) is the second most common type of cancer in China and the third leading cause of cancer-related death [1,2]. The metastatic status of GC serves a critical role in determining the clinical management of the disease, while it is also considered as a significant factor associated with a poor prognosis and reduced overall survival in patients with GC.

Metastasis, caused by aberrant increased cancer cell motility, promotes the migration or invasion of tumor cells to neighboring tissues and their spread to distant organs. The dynamic reorganization of the cytoskeleton plays a critical biological role in the above process [3,4]. Emerging evidence has suggested that the cytoskeleton serves a significant role in tumor progress [5,6]. Through cytoskeletal reorganization, cancer cells acquire the typical morphological changes needed for active cell movement, including the formation of membrane protrusions at the leading edge and membrane contraction at the rear end. The spatial and temporal regulation of the above process is mediated by multiple cellular signaling pathways, while Rho GTPases are universal components of these signaling pathways [3,7,8]. Rho GTPase acts through its activation or inactivation [9–12]. Rho GTPase activation is regulated by guanine nucleotide exchange factors (GEFs), while it is inactivated by GTPase activating proteins (GAPs) [10–12].

Epithelial-to-mesenchymal transition (EMT) has been widely considered as a process involved in initiating cancer metastasis, which is characterized by the loss of epithelial markers and the acquisition of mesenchymal ones [13–17]. EMT is mediated by several transcriptional repressors that target the E-box sequences within the promoter region of E-cadherin. E-cadherin is commonly used as a classic marker of epithelial cells and its loss is associated with the onset of EMT [18]. EMT cortical actin cytoskeleton reorganization in cells is considered as cytoskeletal dynamics and cell elongation directional movement [19,20]. It has been reported that actin‑rich invadopodia exert a proteolytic function in extracellular matrix degradation, thus facilitating cell migration and invasion [19,21,22]. It has been also suggested that during EMT, Rho GTPases regulate F-actin dynamics and control F-actin rearrangement. A previous study showed that RhoA promoted the formation of actin stress fibers, whereas Rac1 and Cdc42 promoted the formation of lamellipodia and filopodia [19]. Additionally, another study suggested that Rho‑associated kinase, LIM kinase and cofilin could also act as downstream molecules when Rho GTPases were activated [19].

A previous study from our laboratory revealed that never in mitosis gene A-related kinase 9 (NEK9) could regulate call metastasis via phosphorylating ARHGEF2, a significant GEF targeting RhoA activation factor [23]. More specifically, the results showed that ARHGAP35 was a candidate target of NEK9. Although further experiments revealed that ARHGAP35 could not be directly targeted by NEK9, it was still considered to be of interest. The ARHGAP35 gene encodes p190A RhoGAP (p190A), a large GAP, which plays a significant role in cell adhesion, migration and invasion [24–26]. ARHGAP35 was also considered as a potential inhibitor of RhoA and was associated with p120RasGAP (p120) [27]. Another study showed that the association of p190A with p120 was promoted by the phosphorylation of ARHGAP35 at Y1105 [27]. Although the RasGAP/RhoGAP complex could not directly affect the catalytic activity of p190A, it promoted the recruitment of p190 to the plasma membrane to enhance its activity on inhibiting Rho expression [27,28]. To date, the effect of ARHGAP35 on GC has not been explored to the best of our knowledge. Therefore, the current study aimed to investigate the function of ARHGAP35 in GC and the association between ARHGAP35 and E-cadherin in gastric cell cytoskeleton reorganization.

The results of the present study demonstrated that ARHGAP35 could directly affect cytoskeletal reorganization and cell motility in GC cells. In addition, ARHGAP35 could inhibit RhoA activation and regulate cell morphology and motility by modulating cytoskeletal reorganization. ARHGAP35 also preserved the expression levels of E-cadherin and inhibited EMT. Furthermore, ARHGAP35 was downregulated in patients with GC and its expression was further decreased in metastatic GC, thus supporting the tumor suppressor nature of ARHGAP35. Overall, the results indicated that the ARHGAP35/RhoA/E-cadherin axis could be a potential strategy for treating patients with GC.

## 2. Methods

### 2.1 Cell culture

The human GC cell line AGS was purchased from China Infrastructure of Cell Line Resources in September 2013. BGC823 cells were maintained in our laboratory. Cells were cultured in RPMI 1640 medium supplemented with 10% FBS (South America Origin IC-1905; BioCytoSci) and 1% penicillin/streptomycin solution at 37°C in an incubator with 5% CO_2_.

### 2.2 Cell transfection

The small interfering (si)RNA sequences targeting ARHGAP35 were obtained from Shanghai GenePharma Co., Ltd. The sequences used were as follows: For si-ARHGAP35-1, forward, GCAGGAUAUUAUCCCUAUUTT, and reverse, AAUAGGGAUAAUAUAAUGCTT; for si-ARHGAP35-2, forward, GCACCUACCAGACAAUCAUTT, and reverse, AUGAUUGUCUGGUAGGUGCTT. The ARHGAP35 overexpression plasmid was synthesized by VectorBuilder Inc. Cells were transfected with the above plasmids/siRNAs using Lipofectamine® 2000 (Invitrogen; Thermo Fisher Scientific, Inc.) according to the manufacturer’s instructions.

### 2.3 Reverse transcription-quantitative PCR (RT-qPCR)

Total RNA was extracted from GC cells using TRIzol® reagent (Invitrogen; Thermo Fisher Scientific, Inc.) according to the manufacturer’s instructions. Subsequently, RNA was reverse transcribed into cDNA using the Advantage RT-for-PCR Kit (Takara Bio, Inc.). qPCR was performed using the SYBR Premix Pro Taq HS qPCR kit (Hunan Accurate Bio-Medical Co., Ltd.) on the CFX96™ Real-Time PCR Detection system (Bio-Rad Laboratories, Inc.). The relative gene expression levels were analyzed using the 2^−ΔΔCq^ method [23]. The primer sequences used were as follows: For ARHGAP35, forward, AGAAAGAGCCGGTTGGTTCAT, and reverse, AACATAGCCAAAGAGGCCTTACG.

### 2.4 Western blot analysis

Briefly, total proteins were extracted using a radio-immunoprecipitation (RIPA) lysis buffer supplemented with protease and phosphatase inhibitors. Western blot analysis was then performed according to the standard procedures, as previously described. The antibodies used were as follows: Anti-ARHGAP35 (cat. no. 2860), anti-E-cadherin (cat. no. 3195S; both from Cell Signaling Technology, Inc.), anti-RhoA (cat. no. ab187027; Abcam), anti-GTP-RhoA (cat. no. ARH05; Cytoskeleton, Inc.) and anti-β-actin (cat. no. A2228; clone AC-74; MilliporeSigma).

### 2.5 Transwell assays

A total of 4 × 10^4^ cells per group were resuspended in serum-free medium and were then seeded into the top chamber of a Transwell insert (8.0-μm pore size; Corning, Inc.). The lower chamber was filled up with 600 μL 1640 medium containing 20% FBS. For invasion assays, the wells of the Transwell insert were pre-coated with 200 mg/ml Matrigel (BD Bioscience). Transwell assays were performed in triplicate [23]. Images of the invaded or migrated cells were captured at a magnification of 200× under a microscope (Olympus BX51; Olympus Corporation). Finally, cells were counted in five randomly selected fields also under a microscope.

### 2.6 Wound healing assay

Cell wound healing assays were carried out at 0 and 24 hours after injury according to the manufacturer’s instructions. Representative images were captured under a microscope. The assays were performed in triplicates. The width of the wound healing was quantified and compared with the baseline values using ImageJ software (National Institutes of Health).

### 2.7 Tissue microarrays and immunohistochemical (IHC) analysis

Tissue microarrays of GC HStmA180Su03 and HStmAde076 were obtained from Shanghai Outdo Biotech Co. Additionally, another GC microarray, including complete pathological data from 45 GC cases (T14-129), was provided by the Xijing Hospital, Fourth Military Medical University (Xi’an, Shaanxi, China). IHC staining was performed according to the manufacturer’s instructions and the results were evaluated by two independent observers. The arrays were scored for staining intensity and protein expression across the section in a double-blinded manner by two pathologists [23]. The tissues were incubated with anti-ARHGAP35 (cat. no. PA1939; AntiProtech, Inc.) and E-cadherin (cat. no. 3195S; Cell Signaling Technology, Inc.) at 4°C overnight according to the manufacturer’s instructions.

### 2.8 Immunofluorescence analysis (IF)

For IF analysis, AGS and BGC823 cells were fixed with 4% paraformaldehyde for 20 minutes at room temperature and were then washed twice with PBS. Subsequently, cells were incubated with rabbit anti-E-cadherin (cat. no. 3195S; Cell Signaling Technology, Inc.) primary antibody at 4°C overnight. The following day, cells were washed thrice with sterile PBS and were then incubated with a conjugated anti-mouse IgG H&L (Alexa Fluor 488; cat. no. ab150113; Abcam) secondary antibody at room temperature for 1 hour. IF images were captured under a confocal microscope (Nikon A1 Plus; Nikon Corporation).

### 2.9 Cytoskeleton staining

Cytoskeleton staining was performed in constructed cell lines using rhodamine phalloidin staining (Cytoskeleton, Inc.) according to the manufacturer’s instructions. Images of the stained were captured under a confocal microscope (Nikon A1 Plus; Nikon Corporation).

### 2.10 Statistical analysis

All statistical analyses were carried out using GraphPad Prism (GraphPad Software, Inc.). One-sided or two-sided statistical tests were applied. The differences between two groups were assessed using Student’s t-test, while those among multiple groups were compared using ANOVA test. The survival rates were determined using the Kaplan-Meier method. Spearman’s correlation analysis was performed to investigate the correlations between different factors based on normality test (r, p). *P* < 0.05 was considered to indicate a statistically significant difference.

## 3. Results

### 3.1 ARHGAP35 is downregulated in human GC tissues and its expression is associated with poor prognosis

To investigate the effect of ARHGAP35 on the clinical outcome and progression of patients with GC, the expression levels of ARHGAP35 were detected in GC tissue microarrays by IHC staining. The results showed that compared with the adjacent non-cancerous tissues, ARHGAP35 was significantly downregulated in GC tissues (Figures 1A_1_-A_2_). The expression levels of ARHGAP35 were also associated with GC progression. Therefore, the decreased expression levels of ARHGAP35 were associated with advanced tumor-nodule-metastasis (TNM) staging (Table 1). In addition, the staining intensity and extent of ARHGAP35 expression was significantly reduced in GC tissues compared with distant metastatic tissues (Figures 1(b-c)). Survival analysis of 114 patients with GC revealed that decreased ARHGAP35 expression was associated with poor prognosis (Figure 1(d)).

**Figure 1.** ARHGAP35 is downregulated in primary GC and metastatic tissues. a_1_-a_2_, The expression levels of ARHGAP35 were determined in GC tissue microarrays by immunohistochemistry. b-c, The expression score of ARHGAP35 in GC, metastatic GC and adjacent normal tissues is shown. **P < 0.05 and ***P < 0.001. d. The overall survival of patients with GC according to their ARHGAP35 expression levels was estimated by Kaplan-Meier analysis. ARHGAP35, Rho GTPase‑activating protein 35; GC, gastric cancer.

**Table 1.** Correlation between ARHGAP35 expression and clinicopathological parameters in GC

Clinicopathological	Total		ARHGAP35 expression		
			Weak expression (-~+)	Strong Positive(++~+++)	*P* value
Variables	(n = 83)		(n = 48)	(n = 35)	
Gender	Male	53	32	21	0.7412
	Female	30	17	13	
Age(y)	≤ 70	51	32	19	0.0902
	> 70	32	14	18	
classification	I+II	15	7	8	0.7362
	III+IV	68	35	33	
T stage	T1+T2	7	1	6	0.0284
	T3+T4	78	48	30	
N stage	N0+N1	32	15	17	0.0307
	N2+N3	51	36	15	
AJCC stage	stage1+2	29	16	13	0.0484
	stage3+4	52	17	35	

### 3.2 ARHGAP35 regulates the migration and invasion of GC cells

Since ARHGAP35 was associated with GC metastasis, the current study explored whether ARHGAP35 could directly affect cell motility. Therefore, an *in vitro* stable ARHGAP35 overexpression or knockdown GC cell model was established in BGC823 and AGS cells (Figures 2(a-b)). Transwell assays demonstrated that ARHGAP35 knockdown in BGC823 and AGS cells attenuated cell migration and invasion. By contrast, ARHGAP35 overexpression exhibited the opposite effect in GC cells (Figures 2(c-d)). Furthermore, the wound healing assays revealed that ARHGAP35 silencing notably accelerated wound closure, while ectopic ARHGAP35 expression delayed the wound healing process (Figures 2(e-f)).

**Figure 2.** ARHGAP35 regulates GC cell motility *in vitro*. a-b, The mRNA and protein expression levels of ARHGAP35 in BGC823 and AGS cells were determined by western blot analysis and reverse transcription-quantitative PCR. *P < 0.05 and **P < 0.01. c-d, The migration and invasion capacities of ARHGAP35-depleted or -overexpressing GC cells were assessed by Transwell assays. d-f. The width of the wound was quantified by cell wound healing assay. **P < 0.01 and ***P < 0.001. ARHGAP35, Rho GTPase‑activating protein 35.

### 3.3 ARHGAP35 regulates cytoskeleton reorganization and EMT via targeting RhoA and E-cadherin

Emerging evidence has suggested that cytoskeletal reorganization and morphological changes are the basis for cell movement. As shown in Figure 3(a), ARHGAP35 knockdown resulted in a spindle-like cell shape, while a number of protrusions were observed at the edge of GC cells in each group, thus indicating the formation of filament- or sheet-shaped pseudopodia. Conversely, ARHGAP35 overexpression exhibited the opposite effect (Figure 3(b)). These findings suggested that cytoskeletal reorganization could be precisely regulated by Rho-GTPases. Furthermore, increased expression of GTP-RhoA was found in ARHGAP35-depleted GC cells (Figure 3(c)), thus resulting in a stronger transition of RhoA from its inactive into an active stage. By contrast, ARHGAP35 overexpression resulted in GTP-RhoA downregulation (Figure 3(c)).

**Figure 3.** ARHGAP35 regulates cytoskeletal reorganization and epithelial-to-mesenchymal transition by targeting RhoA and E-cadherin, respectively. a-b, GC cell cytoskeleton staining was performed using phalloidin. c, The protein expression levels of RhoA and GTP-RhoA were detected by western blot analysis. d, The protein expression levels of e-cadherin were determined in ARHGAP35-depleted or -overexpressing GC cells using western blot analysis. e-f: The expression of the epithelial marker, e-cadherin, in GC cells was assessed by immunofluorescence staining. ARHGAP35, Rho GTPase‑activating protein 35; GC, gastric cancer.

EMT also serves a significant role in cancer metastasis and is characterized by morphological changes resulting from cytoskeletal reorganization. Therefore, in the present study the expression levels of E-cadherin were detected by western blot analysis and IF staining. The results demonstrated that ARHGAP35 overexpression upregulated E-cadherin, thus indicating EMT reversion. By contrast, ARHGAP35 silencing had the opposite effect on EMT via suppressing E-cadherin expression (Figures 3(d-f)).

### 3.4 ARHGAP35 and E-cadherin are simultaneously downregulated in GC metastatic tissues and are associated with a poor prognosis in patients with GC

To explore the effects of ARHGAP35 and E-cadherin expression in human GC tissues on clinical outcomes, their expression levels were assessed in two GC tissue microarrays by IHC. As shown in Figures 4(a-b), a positive correlation between ARHGAP35 and E-cadherin expression was observed. Based on staining intensity and the extent of ARHGAP35 and E-cadherin expression, the results revealed that compared with the corresponding non-cancerous tissues, the expression levels of both proteins were significantly reduced in GC tissues (Figure 4(c)). Similarly, the expression levels of ARHGAP35 and E-cadherin were notably attenuated in metastatic GC tissues compared with GC tissues (Figure 4(c)). Furthermore, the decreased E-cadherin expression levels were associated with reduced overall survival and the combination of both proteins exhibited an enhanced capacity on distinguishing GC patients with different prognosis (Figures 4(d-e)).

**Figure 4.** Simultaneous ARHGAP35 and E-cadherin downregulation is associated with poor prognosis in patients with GC. a-b-, The expression levels of ARHGAP35 and E-cadherin were determined in tissue microarrays by immunohistochemistry. c, A positive association between the expression of ARHGAP35 and E-cadherin was revealed in GC. d, E-cadherin downregulation was associated with poor prognosis in patients with GC. e, The association between ARHGAP35/E-cadherin co-expression and overall survival in patients with GC is shown. ARHGAP35, Rho GTPase‑activating protein 35; GC, gastric cancer.

In summary, the current study reported a novel signaling pathway involved in GC metastasis. ARHGAP35 could directly regulate cell morphology and motility via affecting cytoskeleton reorganization and EMT through targeting RhoA and E-cadherin, respectively. Additionally, the results showed that ARHGAP35 was downregulated in patients with GC and its expression was further reduced in metastatic GC tissues. The aforementioned findings supported the possible role of ARHGAP35 as a tumor suppressor factor. Overall, the results suggested that the ARHGAP35/RhoA/E-cadherin axis could serve as a potential approach for treating metastatic GC.

## 4. Discussion

The results of the current study suggested that ARHGAP35 could act as negative regulator in GC metastasis. ARHGAP35 could inhibit the activation of RhoA via directly targeting RhoA, thus resulting in cytoskeletal reorganization. In addition, ARHGAP35 also induced the expression of E-cadherin and antagonized the occurrence of EMT. Furthermore, the potential roles of ARHGAP35 were further assessed by clinical evaluation in GC specimen. Therefore, the analysis revealed that ARHGAP35 was downregulated in metastatic GC and it was associated with the overall survival of patients with GC. Overall, this was the first study systematically exploring the effects of ARHGAP35 in GC, thus supporting its universal role in cancer metastasis.

ARHGAP35, a multidomain RhoGAP, contains N-terminal pseudo GTPase and C-terminal RhoGAP domains [29]. There is a flexible region between these domains that is commonly phosphorylated at Tyr-1087 and Tyr-1105 residues [29]. The above post-translational modification is responsible for the recruitment of ARHGAP35 to the plasma membrane where it properly regulates Rho cascades. The phosphorylation of ARHGAP35 plays a significant role in its interaction with p120RasGAP at plasma membrane [29,30]. In a previous study from our laboratory focusing on the function of NEK9, a serine-threonine kinase, phosphorylomics were employed to systemically analyze its targets. Therefore, the analysis revealed that ARHGAP35 was a potential effector of NEK9 [23]. Although ARHGAP35 was not phosphorylated by NEK9, it was still necessary to explore the upstreaming kinase targeting ARHGAP35. In breast cancer, a breast cancer kinase could phosphorylate ARHGAP35, which in turn could regulate Rho and Ras and promote cancer cell growth, migration and invasion [27]. In addition, another study suggested that ARHGAP35 was a substrate of glycogen synthase kinase‑3 and could be involved in polarized cell migration. Therefore, these findings suggested that ARHGAP35 could be phosphorylated by different kinases in a tissue- or organ-specific manner. Therefore, screening and validating the upstream kinases of ARHGAP35 could be a promising strategy for broadening the current understanding on its effects.

The activation of RhoGAP is considered as the key function of ARHGAP35. By binding to RhoA, ARHGAP35 promotes the accumulation of GDP-bound RhoA and reduces that of GTP-bound RhoA. The above effect of ARHGAP35 was confirmed in the current study, thus supporting its universal and fundamental role in regulating cell motility. RhoA inactivation is directly involved in the morphological changes of cancer cells, mainly mediated by cytoskeleton reorganization. Herein, the density of actin bundles was significantly increased in ARHGAP35-depleted GC cells. The protrusions along the leading edge of the spindle-shaped GC cancer cells indicated the active formation of pseudopodia, a direct evidence of active cell movement.

In addition to regulating RhoA activation, ARHGAP35 was also found to promote E-cadherin expression, thus indicating EMT reversion. Since EMT is considered to be a significant factor during the initiation of cancer metastasis, reversing EMT could be another mechanism of ARHGAP35 to suppress GC metastasis. Actually, a previous study also highlighted the intrinsic association of ARHGAP35 and E-cadherin expression in the regulation of tumor growth [27]. Additionally, another study showed that ARHGAP35 could promote contact inhibition of proliferation via activating large tumor suppressor (LATS) kinases and phosphorylating the proto-oncogenic transcriptional co-activator Yes‑associated protein [31]. Therefore, ARHGAP35 induced E-cadherin expression, which in turn enhanced the ARHGAP35-mediated activation of LATS. Although the above findings strongly suggested that the ARHGAP35-triggered regulation of E-cadherin could play a critical role in cancer development, their clinical significance has not been systematically investigated. Therefore, in the present study the expression levels of both ARHGAP35 and E-cadherin were detected in multiple sets of GC tissue microarrays. The results showed that the intensity of ARHGAP35 was positively associated with that of E-cadherin, while a gradual and simultaneous reduction in their expression levels was obtained in primary and metastatic GC tissues compared with non-cancerous ones. The prognostic value of the combined ARHGAP35 and E-cadherin expression was also confirmed in the current study, since loss of their expression was associated with reduced overall survival in patients with GC. A previous study demonstrated that cadherin-induced entosis was associated with ARHGAP35 activity-dependent polarized distribution in human breast cancer cells. Additionally, a previous study from our laboratory suggested that ARHGAP35 could directly regulate cell cytoskeleton reorganization via activating RhoA and could suppress GC cell metastasis via upregulating E-cadherin [32]. The above findings from clinical specimens highlighted the potential use of ARHGAP35 and E-cadherin in clinical practice, thus verifying the clinical significance and value of the current study.

## Conclusion

The current study suggested that ARHGAP35 could inhibit the activation of RhoA and suppress GC metastasis by promoting cytoskeleton reorganization. In addition, ARHGAP35 overexpression downregulated E-cadherin, thus indicating EMT reversion. The expression of both ARHGAP35 and E-cadherin was associated with the metastatic status of GC and their combination could therefore serve as a potential strategy for evaluating the development of GC. The above findings prompted us to further investigate in future studies the molecular mechanisms underlying the effect of ARHGAP35 on inhibiting the progression of GC such as the activation of the membrane-associated periodic skeleton or receptor tyrosine kinase pathways.

## Abbreviations

GC: Gastric cancer; GEFs: Guanine nucleotide exchange factors; EMT: Epithelial-to-mesenchymal transition; ROCK: Rho‑associated kinase; LIMK: LIM kinase; NIMA: Never in mitosis gene; RIPA: Radioimmunoprecipitation; IHC: Immunohistochemical; IF: Immunofluorescence analysis
